The article "Coracoid Abnormalities and Their Relationship with Glenohumeral Deformities in Children with Obstetric Brachial Plexus Injury" was published in 2010. Journal: BMC Musculoskelet Disord.

# Coracoid Abnormalities and Their Relationship with Glenohumeral Deformities in Children with Obstetric Brachial Plexus Injury

**DOI:** 10.1186/1471-2474-11-237

**Published:** 2010-10-13

**Authors:** Rahul K Nath, Faiz Mahmooduddin, Xiaomei Liu, Melissa J Wentz, Andrea D Humphries

**Affiliations:** 1 Texas Nerve and Paralysis Institute, 6400 Fannin Street, Suite 2420, Houston, TX, 77030, USA

## Abstract

**Background:**

Patients with incomplete recovery from obstetric brachial plexus injury (OBPI) usually develop secondary muscle imbalances and bone deformities at the shoulder joint. Considerable efforts have been made to characterize and correct the glenohumeral deformities, and relatively less emphasis has been placed on the more subtle ones, such as those of the coracoid process. The purpose of this retrospective study is to determine the relationship between coracoid abnormalities and glenohumeral deformities in OBPI patients. We hypothesize that coracoscapular angles and distances, as well as coracohumeral distances, diminish with increasing glenohumeral deformity, whereas coracoid overlap will increase.

**Methods:**

39 patients (age range: 2-13 years, average: 4.7 years), with deformities secondary to OBPI were included in this study. Parameters for quantifying coracoid abnormalities (coracoscapular angle, coracoid overlap, coracohumeral distance, and coracoscapular distance) and shoulder deformities (posterior subluxation and glenoid retroversion) were measured on CT images from these patients before any surgical intervention. Paired Student t-tests and Pearson correlations were used to analyze different parameters.

**Results:**

Significant differences between affected and contralateral shoulders were found for all coracoid and shoulder deformity parameters. Percent of humeral head anterior to scapular line (PHHA), glenoid version, coracoscapular angles, and coracoscapular and coracohumeral distances were significantly lower for affected shoulders compared to contralateral ones. Coracoid overlap was significantly higher for affected sides compared to contralateral sides. Significant and positive correlations were found between coracoscapular distances and glenohumeral parameters (PHHA and version), as well as between coracoscapular angles and glenohumeral parameters, for affected shoulders. Moderate and positive correlations existed between coracoid overlap and glenohumeral parameters for affected shoulders. On the contrary, all correlations between the coracoid and glenohumeral parameters for contralateral shoulders were only moderate or relatively low.

**Conclusions:**

These results indicate that the spatial orientation of the coracoid process differs significantly between affected and contralateral shoulders, and it is highly correlated with the glenohumeral deformity. With the progression of glenohumeral deformity, the coracoid process protrudes more caudally and follows the subluxation of the humeral head which may interfere with the success of repositioning the posteriorly subluxed humeral head anteriorly to articulate with the glenoid properly.

## Background

Obstetric brachial plexus injury commonly involves injury to C5 and C6 nerve roots. Most patients recover spontaneously within the first three months of life. Patients without adequate recovery of neurological function will develop secondary muscle imbalances and bone deformities at the shoulder joint, which are the major causes of long-term morbidity in this patient population [1-4]. Characteristic anatomical changes of the shoulder joint include glenohumeral dysplasia and dislocation and posterior subluxation of the humeral head. Considerable efforts have been made to characterize and correct the glenohumeral deformities in patients with obstetric brachial plexus injury, but relatively less emphasis has been placed on the more subtle ones, such as those of coracoid process.

Abnormal growth of the coracoid process has been observed in patients with obstetric brachial plexus injury [1,5-9]. Birch [1] reported that in 166 patients with secondary bone deformities, 90 had moderate coracoid overgrowth and 36 had severe coracoid overgrowth. Kambhampati *et al. *[7] developed a grading system to classify the deformity of the coracoid. Upon intra-operative observation in 183 patients, they found that almost 57% of the patients had grade 1 and 31% had grade 2 coracoid deformity (grade 0 means a normal coracoid, grade 1 means a moderately deformed coracoid with the tip at the level of capital physis, and grade 2 means a severely deformed coracoid with the tip below the level of capital physis). Despite these obvious abnormalities observed in the coracoid process, there are few studies correlating these abnormalities with glenohumeral deformities commonly occurring in this patient population. Soldado et al conducted a study demonstrating a relationship between the coracoid and glenoid during shoulder development. A correlation was found between a decrease in glenoid physeal angle (glenoid retroversion) with a simultaneous increase in the coracoid physeal angle (coracoid retroversion) and a decrease in the coracoscapular distance [6].

The purpose of this retrospective study is to determine the relationship between coracoid abnormalities and glenohumeral deformities (posterior subluxation and glenoid retroversion) in OBPI patients. We hypothesize that coracoscapular angles and distances, as well as coracohumeral distances, diminish with increasing glenohumeral deformity, whereas coracoid overlap will increase.

This study has clinical relevance in that its results can potentially help in pre-operative planning of surgical procedures to correct glenohumeral deformites of OBPI patients. Surgical intervention usually involves repositioning the posteriorly subluxed humeral head anteriorly to articulate with the glenoid properly. However, the abnormal spatial orientation of the coracoid process can interfere with the success of this procedure. Therefore, it is important to understand the spatial relationship of the coracoid process with the shoulder joint prior to surgical treatments. Understanding a possible relationship between the coracoid and glenohumeral deformity can assist in the success of surgical procedures such as open reduction or arthroscopic anterior glenohumeral capsule release.

## Methods

The parents of the patients that were a part of this study have given informed consent for their children to be included in the study and for the photos to be published in scientific journals. Our research is not federally funded; therefore, there is no approval from institutional review board needed for our research. All of our research and studies on human subjects are in compliance with the Declaration of Helsinki.

Inclusion criteria for patients to be a part of this study was as follows:

1. Age > = 2 years (at which the coracoid ossification center expands and the tip of the coracoid process is clearly identifiable [10])

2. Have deformities secondary to OBPI

3. Underwent modified Quad [4] and/or triangle tilt procedures [11]

4. Surgeries occurred from January 2007 to August 2009

5. Had CT images before any surgical intervention was done.

Exclusion criteria was as follows:

1. Age < 2 years

2. No deformities secondary to OBPI

3. Underwent other operations instead of modified Quad or triangle tilt

4. Surgeries occurred earlier than January 2007 or after August 2009

5. No pre-operative CT images available

Thirty nine patients met the inclusion criteria. Data was retrospectively collected on pre-operative CT images of both affected and contralateral shoulders in order to represent the original anatomy of bony structures. These 39 patients had varied degree of initial nerve injury which involved C5-C6, C5-C6-C7, or C5-T1 roots. There were 12 left-sided and 27 right-sided injuries. There were 15 males and 24 females, ranging in age from 2-13 years and with an average age of 4.7 years and median age of 4 years at the time of pre-operative CT exams.

The parameters used to assess coracoid abnormalities in this study included coracoscapular angle, coracoid overlap, coracohumeral distance, and coracoscapular distance, which were measured on axial CT images taken from the patients pre-operatively. These axial images clearly showed the center of the humeral head, the glenoid portion articulating with the humeral head, and the tip of the coracoid process. Depending on the position of the coracoid tip, the level of axial CT image chosen may not be the same for each patient. The measurement of the coracoscapular angle was based on a scapular line "a" that was constructed to connect the midpoint between the most anterior and posterior portion of the glenoid labrum to the medial margin of the scapula, and a line "b" that started at the most anterior portion of the glenoid labrum and ran tangentially to the most prominent aspect of the coracoid tip (Figure 1). The angle between lines "a" and "b" was defined as the coracoscapular angle, which is different from the angles measured from previous studies [6,12] and is considered to be more representative for the relationship between the coracoid process and the glenohumeral joint in patients with obstetric brachial plexus injury. The coracoid overlap was measured as the perpendicular distance from the most lateral aspect of the coracoid tip to the plane of the glenoid (represented as line "c" on Figure 1) that went through the most anterior and posterior portion of the glenoid labrum representing the distance by which the coracoid overlapped the glenoid plane [12]. The coracohumeral distance was adapted from Gerber *et al. *[12] due to the incomplete ossification of the humeral head and the hypoplasia from the brachial plexus injury. It was defined as the distance from the tip of the coracoid process to the calculated center of the humeral head that was visible in CT images, instead of the subchondral bone of the humeral head (Figure 1). The coracoscapular distance was measured as the perpendicular distance from the most lateral aspect of the coracoid tip to the scapular line as previously described [6].

**Figure 1:** **Representative axial CT image of the affected shoulder from a patient with obstetric brachial plexus injury**. Line "a" is the scapular line. Line "b" starts at the most anterior portion of the glenoid labrum and runs tangentially to the most prominent aspect of the coracoid tip. Line "c" represents the glenoid plane. Angle "A" formed between lines "a" and "b" is the coracoscapular angle. C-G represents the distance of coracoid overlap. C-HH represents the coracohumeral distance. C-S represents the coracoscapular distance.

The glenohumeral deformity parameters measured in this study were posterior subluxation of the humeral head and glenoid retroversion. On axial CT images (which may not be the same as those used for measuring coracoid parameters due to the different position of the coracoid tip) representing the exact relationship of the humeral head and glenoid fossa, posterior subluxation was quantified as the percent of the humeral head anterior to the scapular line (PHHA) according to Waters *et al. *[5] but using a circle to represent anterior and posterior margins of the humeral head because of the incomplete ossification in young patients, and version was quantified as the glenoscapular angle subtracted by 90° modified from Friedman *et al. *[13] using the glenoid surface contacting the humeral head rather than the line connecting anterior and posterior margins (due to the presence of pseudoglenoid in some cases).

All the measurements were performed by trained scientists (XL and MJW) independent of the surgeon and senior author. Graphic software (Universal Desktop Ruler, AVP-Soft.com, Voronezh, Russia) was used for all measurements made on axial CT images. Distance was measured in pixels, and converted into standard length units as millimeters (mm).

The mean and standard error of the mean were calculated for each measured parameter. The paired Student's t-test was conducted to determine any significant difference between affected and contralateral shoulders for each measured parameter. The test of Pearson correlation was also performed to determine the correlations between coracoid and glenohumeral deformity parameters. Results were considered statistically significant at *p *< 0.05 level. All statistical analyses were performed using Analyse-It plugin for Microsoft Excel 2003 software (Leeds, UK).

## Results

Patients included in our study had varying degree of secondary deformities and typically presented with fixed medial rotation contracture and scapular deformity with coracoids that were elongated and hooked in appearance on the affected shoulders as visible in CT images (Figure 2).

**Figure 2:** **Panel a: A patient with residual brachial plexus injury typically presented with fixed medial rotation contracture of the affected shoulder**. Panel b: A 3D CT image from the same patient showing elevated scapula and elongated coracoid process (directed more towards the humeral head) of the affected shoulder.

### Summary of results for measurement parameters

Mean and standard error of the mean calculated for each measurement parameter are shown in Figure 3, as well as *p *values from paired Student t-test comparing each measurement parameter between affected and contralateral shoulders.

**Figure 3:** **Statistical comparison of posterior subluxation, glenoid version, coracoscapular angle, coracoid overlap, coracoscapular distance, and coracohumeral distance between the affected and contralateral shoulders**. ***: *p *< 0.001.

The average value of PHHA was 25% (2) for the affected shoulders and 43% (2) for the contralateral shoulders. The average value of glenoid version was -23° (2) for the affected sides and -5° (1) for the contralateral sides. The values of PHHA and glenoid version were significantly lower for the affected shoulders compared to those for the contralateral shoulders (*p *< 0.0001) as shown in Figure 3.

Values of the coracoscapular angle, the angle between the scapular line and the line that connected the most anterior portion of the glenoid labrum and the most prominent aspect of the coracoid tip, were significantly lower for the affected shoulders compared to those for the contralateral shoulders (25° (2) vs. 51° (1), *p *< 0.0001, Figure 3). Similarly, values of the coracoscapular distance, the perpendicular distance from the most prominent aspect of the coracoid tip to the scapular line, were significantly lower for the affected sides compared to those for the contralateral sides (16.0 mm (0.6) vs. 21.5 mm (0.8), *p *< 0.0001, Figure 3). Values of the coracohumeral distance, measured as the distance from the most prominent aspect of the coracoid tip to the calculated center of the ossified humeral head visible on the axial CT image, were significantly lower for the affected shoulders compared to those for the contralateral ones (24.3 mm (0.7) vs. 26.2 mm (0.7), *p *= 0.005, Figure 3). On the contrary, values of the coracoid overlap, presented as the perpendicular distance by which the coracoid overlapped the plane of the glenoid, were significantly higher for the affected sides compared to those for the contralateral sides (11.1 mm (0.7) vs. 8.5 mm (0.4), *p *= 0.0008, Figure 3).

### Correlations between coracoid and glenohumeral deformity parameters for affected and contralateral shoulders

The Pearson correlation was conducted between coracoid and glenohumeral parameters for both affected and contralateral shoulders and results were tabulated in Table 1. Significant and positive correlations were found between coracoscapular angle and glenohumeral parameters (PHHA and version) for the affected shoulders. Similarly, significant and positive correlations were found between coracoscapular distance and glenohumeral parameters (PHHA and version) for the affected shoulders. Moderate and positive correlations existed between coracoid overlap and glenohumeral parameters (PHHA and version) for the affected shoulders. On the contrary, all the correlations between coracoid and glenohumeral parameters for the contralateral shoulders were only moderate or relatively low.

**Table 1:** Correlations between coracoid and glenohumeral parameters for affected and contralateral shoulders

	PHHA		Version	
	
	Affected	Contralateral	Affected	Contralateral
Coracoscapular angle	r = 0.83 (p < 0.0001)	r = 0.53 (p = 0.0008)	r = 0.78 (p < 0.0001)	r = 0.33 (p = 0.0450)
Coracoscapular distance	r = 0.68 (p < 0.0001)	r = 0.58 (p = 0.0002)	r = 0.66 (p < 0.0001)	r = 0.02 (p = 0.9239)
Coracoid overlap	r = 0.42 (p = 0.0075)	r = 0.24 (p = 0.1456)	r = 0.56 (p = 0.0002)	r = 0.13 (p = 0.4284)

## Discussion

We measured glenohumeral and coracoid parameters on CT images and compared results obtained for the affected shoulders to those for the contralateral ones. Significant differences for all measurement parameters were found between the affected and contralateral shoulders, which were consistent with previous studies [6,14,15]. Values of coracoscapular angle, coracoscapular distance and coracohumeral distance were significantly lower for the affected shoulders as compared to those for the contralateral shoulders, whereas values of coracoid overlap were significantly higher for the affected shoulders when compared to those for the contralateral shoulders (Figure 3). These results indicate that the spatial orientation of the coracoid process differs between the affected and contralateral shoulders. Therefore, brachial plexus injury affects not only the glenohumeral joint, but also the coracoid process. Meanwhile, significant and positive correlations between coracoscapular angle and posterior subluxation, coracoscapular angle and version, coracoscapular distance and posterior subluxation, coracoscapular distance and version for the affected shoulders while not for the contralateral shoulders indicate that the coracoid deformity is highly correlated with glenohumeral deformity. The worse the glenohumeral deformity, the smaller the values of coracoscapular angle and coracoscapular distance. A decreased coracoscapular angle and coracoscapular distance mean that the coracoid process protrudes more towards the scapular line and the humeral head. These coracoid abnormalities may be attributed to the tension induced by the medial rotation contracture and/or the posterior subluxation of the humeral head that is placed on the coracoid process [6,16].

Changes in the coracohumeral distance depend on the relative changes in the positions of coracoid tip and humeral head during the progression of glenohumeral deformity. Therefore, the coracohumeral distance could not be simply correlated with glenohumeral parameters as other coracoid parameters did. Multiple effects from both coracoid and glenohumeral parameters should be considered. The average difference in coracohumeral distances between affected and unaffected sides was about 2 mm in this study which is close to 10% of the total coracohumeral distance of the unaffected side. This can potentially be explained by the hypoplasia of the affected scapula, or the SHEAR (scapular hypoplasia, elevation, and rotation) deformity noted in OBPI patients, in which the affected scapula is also nearly 10% smaller than the unaffected scapula [14]. A theoretical explanation of this phenomenon considers the possibility of a constant ratio of coracohumeral distance to scapular size. Movements of the humeral head (internal and external rotation and abduction) all influence the growth and direction of the coracoid. In OBPI, these movements are reduced and humeral head subluxation occurs in addition to the development of the SHEAR deformity. The coracoid may follow the migrating head keeping more or less the same ratio of coracohumeral distance to scapular size.

Our study demonstrates significant correlation between coracoid parameters and glenohumeral deformities in patients with obstetric brachial plexus injury. Shoulders with severe posterior subluxation of the humeral head and glenoid version exhibit shorter coracoscapular distances, smaller coracoscapular angles, and greater coracoid overlap..

With the progression of glenohumeral deformity, the coracoid process protrudes more caudally and follows the subluxation of the humeral head. Effectively, the coracohumeral distance narrows due to the presence of posterior subluxation of the humeral head in the affected shoulders. The coracohumeral distance especially becomes shorter when the shoulder is internally rotated [17]., The coracoid overlap is larger in patients with glenohumeral deformities for reasons similar to those mentioned above. Medial rotation contracture cause posterior subluxation of the humeral head and glenoid version. These factors then influence the growth and direction of the coracoid as the coracoid follows the migrating humeral head. As a result, the coracoid intersects and overlaps the plane of the glenoid.

Surgical intervention is usually required for these patients to correct their glenohumeral deformities by repositioning the posteriorly subluxed humeral head anteriorly to articulate properly with the glenoid. However, the abnormal spatial orientation of the coracoid process can potentially interfere with the success of this procedure. Therefore, it is important to understand the spatial relationship of the coracoid process with the shoulder joint prior to surgical treatments. We recommend that surgical procedures should take into account the abnormal coracoid process. Further studies are needed to evaluate these considerations more thoroughly.

In this study all measurements are performed on CT images; therefore, only bony structures and anatomy may be measured. Future studies using MRI, which may allow for measurements of cartilaginous structures as well, are encouraged. Perhaps more accurate and precise measurements can then be made for coracohumeral and coracoscapular distances, as well as coracoid overlap. This may allow for additional measurements in children with obstetric brachial plexus injuries due to varying ossification of their bony structures.

## Competing interests

The authors declare that they have no competing interests.

## Authors' contributions

RKN conceived the study, participated in the design of the study and revision of the manuscript. FM participated in the analysis and interpretation of the data and revision of the manuscript. XL participated in the design of the study, collection of data, drafting and revision of the manuscript. MJW and ADH participated in the design of the study, collection of data and revision of the manuscript. All authors have read and approved the final manuscript.

## Pre-publication history

The pre-publication history for this paper can be accessed here:

http://www.biomedcentral.com/1471-2474/11/237/prepub
